# Analyzing huge pathology images with open source software

**DOI:** 10.1186/1746-1596-8-92

**Published:** 2013-06-06

**Authors:** Christophe Deroulers, David Ameisen, Mathilde Badoual, Chloé Gerin, Alexandre Granier, Marc Lartaud

**Affiliations:** 1 Univ Paris Diderot, Laboratoire IMNC, UMR 8165 CNRS, Univ Paris-Sud, Orsay F-91405, France; 2 Univ Paris Diderot, Laboratoire de pathologie, Hôpital Saint-Louis APHP, INSERM UMR-S 728, Paris F-75010, France; 3 CNRS, UMR 8165, Laboratoire IMNC, Univ Paris-Sud, Univ Paris Diderot, Orsay F-91405, France; 4 Present address: CNRS, UMR 8148, Laboratoire IDES, Univ Paris-Sud, Orsay F-91405, France; 5 Present address: CNRS, UMR 8608, IPN, Univ Paris-Sud, Orsay F-91405, France; 6 MRI-Montpellier RIO Imaging, CRBM, Montpellier F-34293, France; 7 CIRAD, Montpellier CEDEX 5 F-34398, France

**Keywords:** Digital pathology, Image processing, Virtual slides, Systems biology, ImageJ, NDPI

## Abstract

**Background:**

Digital pathology images are increasingly used both for diagnosis and research, because slide scanners are nowadays broadly available and because the quantitative study of these images yields new insights in systems biology. However, such virtual slides build up a technical challenge since the images occupy often several gigabytes and cannot be fully opened in a computer’s memory. Moreover, there is no standard format. Therefore, most common open source tools such as ImageJ fail at treating them, and the others require expensive hardware while still being prohibitively slow.

**Results:**

We have developed several cross-platform open source software tools to overcome these limitations. The NDPITools provide a way to transform microscopy images initially in the loosely supported NDPI format into one or several standard TIFF files, and to create mosaics (division of huge images into small ones, with or without overlap) in various TIFF and JPEG formats. They can be driven through ImageJ plugins. The LargeTIFFTools achieve similar functionality for huge TIFF images which do not fit into RAM. We test the performance of these tools on several digital slides and compare them, when applicable, to standard software. A statistical study of the cells in a tissue sample from an oligodendroglioma was performed on an average laptop computer to demonstrate the efficiency of the tools.

**Conclusions:**

Our open source software enables dealing with huge images with standard software on average computers. They are cross-platform, independent of proprietary libraries and very modular, allowing them to be used in other open source projects. They have excellent performance in terms of execution speed and RAM requirements. They open promising perspectives both to the clinician who wants to study a single slide and to the research team or data centre who do image analysis of many slides on a computer cluster.

**Virtual slides:**

The virtual slide(s) for this article can be found here:

http://www.diagnosticpathology.diagnomx.eu/vs/5955513929846272

## Background

Virtual microscopy has become routinely used over the last few years for the transmission of pathology images (the so-called virtual slides), for both telepathology and teaching [1,2]. In more and more hospitals, virtual slides are even attached to the patient’s file [3,4]. They have also a great potential for research, especially in the context of multidisciplinary projects involving e.g. mathematicians and clinicians who do not work at the same location. Quantitative histology is a promising new field, involving computer-based morphometry or statistical analysis of tissues [5-9]. A growing number of works report the pertinence of such images for diagnosis and classification of diseases, e.g. tumours [10-14]. Databases of clinical cases [15] will include more and more digitized tissue images. This growing use of virtual microscopy is accompanied by the development of integrated image analysis systems offering both virtual slide scanning and automatic image analysis, which makes integration into the daily practice of pathologists easier. See Ref. [16] for a review of some of these systems.

Modern slide scanners produce high magnification microscopy images of excellent quality [1], for instance at the so-called “40x” magnification. They allow much better visualization and analysis than lower magnification images. As an example, Figure 1 shows two portions of a slide at different magnifications, 10x and 40x. The benefit of the high magnification for both diagnosis and automated image analysis is clear. For instance, the state of the chromatin inside the nucleus and the cell morphology, better seen at high magnification, are essential to help the clinician distinguish tumorous and non-tumorous cells. An accurate, non-pixelated determination of the perimeters of the cell nuclei is needed for morphometry and statistics.

**Figure 1:** **A sample slide.** (**a**): macroscopic view of the whole slide (the black rectangle on the left is 1x2 cm). (**b,c**): Influence of the magnification on the quality of results. (**b**): a portion of the slide scanned at magnification level 10x. The white contours show the result of an automatic detection of the dark cell nuclei with the ImageJ software. A significant fraction of the cell nuclei is missed and the contours are rather pixelated. (**c**): the same portion of the slide scanned at magnification 40x. The white contours show the result of the same automatic detection. Almost all cell nuclei are detected and the shapes of the contours are much more precise. Scale bar: 4 *μ*m.

However, this technique involves the manipulation of huge images (of the order of 10 billions of pixels for a full-size slide at magnification 40x with a single focus level) for which the approach taken by most standard software, loading and decompressing the full image into RAM, is impossible (a single slice of a full-size slide needs of the order of 30 GiB of RAM). As a result, standard open-source software such as ImageJ [17], ImageMagick [18] or GraphicsMagick [19] completely fails or is prohibitively slow when used on these images. Of course, commercially available software exists [16], but it is usually quite expensive, and very often restricted to a single operating system. It uses proprietary source code, which is a problem if one wants to control or check the algorithms and their parameters when doing image analysis for research.

In addition, many automated microscopes or slide scanners store the images which they produce into proprietary or poorly documented file formats, and the software provided by vendors is often specific to some operating system. This leads to several concerns. First, it makes research based on digital pathology technically more difficult. Even when a project is led on a single site, one has often to use clusters of computers to achieve large-scale studies of many full-size slides from several patients [20]. Since clusters of computers are typically run by open source software such as Linux, pathology images stored in non-standard file formats are a problem. Furthermore, research projects are now commonly performed in parallel in several sites, not to say in several countries, thanks to technology such as Grid [21], and there is ongoing efforts towards the interoperability of information systems used in pathology [3,22]. Second, proprietary formats may hinder the development of shared clinical databases [15] and access of the general public to knowledge, whereas the citizen should receive benefit of public investments. Finally, they may also raise financial concerns and conflicts of interest [23].

There have been recent attempts to define open, documented, vendor-independent software [24,25], which partly address this problem. However, very large images stored in the NDPI file format produced by some slide scanners manufactured by Hamamatsu, such as the NanoZoomer, are not yet fully supported by such software. For instance, LOCI Bio-Formats [25] is presently unable to open images, one dimension of which is larger than 65k, and does not deal properly with NDPI files of more than 4 GiB. OpenSlide [24] does not currently support the NDPI format. NDPI-Splitter [26] needs to be run on Windows and depends on a proprietary library.

To address these problems, we have developed open source tools which achieve two main goals: reading and converting images in the NDPI file format into standard open formats such as TIFF, and splitting a huge image, without decompressing it entirely into RAM, into a *mosaic* of much smaller pieces (tiles), each of which can be easily opened or processed by standard software. All this is realized with high treatment speed on all platforms.

## Implementation

### Overview

The main software is implemented in the C programming language as separate, command-line driven executables. It is independent of any proprietary library. This ensures portability on a large number of platforms (we have tested several versions of Mac OS X, Linux and Windows), modularity and ease of integration into scripts or other software projects.

It is complemented by a set of plugins for the public domain software ImageJ [17], implemented in Java, which call the main executables in an automatic way to enable an interactive use.

The LargeTIFFTools and NDPITools are based on the open source TIFF [27] and JPEG [28] or libjpeg-turbo [29] libraries. The NDPITools plugins for ImageJ are based on the Java API of ImageJ [17,30] and on the open source software Image-IO [31], and use the Java Advanced Imaging 1.1.3 library [32].

### Basic functions

The basic functions are the following. They can be performed even on a computer with a modest amount of RAM (see below the “Performance” discussion). 

1. splitting a tiled TIFF file into multiple TIFF files, one for each of the tiles (tiffsplittiles program);

2. extracting (“cropping”) quickly a given rectangle of a supposedly tiled TIFF file into a TIFF or JPEG file (tifffastcrop program);

3. splitting one or several TIFF file(s), possibly very large, into mosaic(s), without fully decompressing them in memory (tiffmakemosaic program);

4. converting a NDPI file into a standard multiple-image TIFF file, tiled if necessary, using upon request the BigTIFF format introduced in version 4.0.0 of the TIFF library [27,33,34], and encoding magnification and focus levels as TIFF “image description” fields (ndpi2tiff program);

5. creating a standard TIFF file for all or part of the magnification levels and focus levels present in the given NDPI file (the user can ask for specific magnification and focus levels and for a specific rectangular region of the image), and, upon request, creating a mosaic for each image which doesn’t fit into RAM or for all images (ndpisplit program). The names of the created files are built on the name of the source file and incorporate the magnification and focus levels (and, in the case of mosaic pieces, the coordinates inside the mosaic).

### Mosaics

A mosaic is a set of TIFF or JPEG files (the *pieces*) which would reproduce the original image if reassembled together, but of manageable size by standard software. The user can either specify the maximum amount of RAM which a mosaic piece should need to be uncompressed (default: 1024 MiB), or directly specify the size of each piece. In the first case, the size of each piece is determined by the software. A given amount of overlap between mosaic pieces can be requested, either in pixels or as a percentage of the image size. This is useful e.g. for cell counting, not to miss cells which lie on the limit between two adjacent pieces.

### Usage

#### Standalone

Our tools can be used through the command line (POSIX-like shell or Windows command interpreter), and therefore can be very easily integrated into scripts or other programs. Depending on the tool, the paths and file names of one or several files, in NDPI or TIFF format, have to be provided. Options can be added with their arguments on the command line to modify the behavior of the programs from its default. They are explained in the messages printed by the programs run without arguments, in Unix-style man pages, and on the web pages of the project (see below in the *Availability and requirements* Section).

Under the Windows OS, one can click-and-drag the NDPI file icon onto the icon of ndpi2tiff or ndpisplit. We provide precompiled binaries where frequently-used options are turned on by default: e.g. ndpisplit-mJ.exe produces a mosaic in JPEG format as with option -mJ. The conversion result or mosaic can be found in the same directory as the original NDPI image.

#### ImageJ integration

In addition to command line use, the ndpisplit program can be driven through the NDPITools plugins in ImageJ with a point-and-click interface, so that previewing the content of a NDPI file at low resolution, selecting a portion, extracting it at high resolution and finally opening it in ImageJ to apply further treatments can be done in an easy and graphical way. Figure 2 shows a screen shot of ImageJ 1.47 m after extraction of a rectangular zone from a NDPI file. Figure 3 explains what happens when the NDPI file contains several levels of focalization: the preview image is displayed as a stack.

**Figure 2:** **A typical session using ImageJ and the NDPITools plugins.** A NDPI file has been opened with the NDPITools plugins and it is displayed as a preview image (image at largest resolution which still fits into the computer’s screen) — top window. A rectangular region has been selected and extracted as a TIFF image, then opened — bottom window.

**Figure 3:** **Preview image of a NDPI file with several focalization levels in ImageJ.** The NDPI file 08.ndpi contains images at 5 different focalization levels. Therefore, its preview image is displayed as a stack of 5 images.

When producing a mosaic, the user can request that pieces be JPEG files. Since the File > Open command of versions 1.x of ImageJ is unable to open TIFF files with JPEG compression (one has to use plugins), this is way to produce mosaics which can be opened by click-and-drag onto the window or icon of ImageJ while still saving disk space thanks to efficient compression. Figure 4 shows how the mosaic production options can be set inside ImageJ through the NDPITools plugins.

**Figure 4:** **Dialog box for customized extraction in ImageJ from an NDPI file with production of a mosaic.** The dialog box shows some options which can be customized while producing a mosaic from a rectangular selection of a NDPI file preview image (here, using the file previewed in Figure 3).

## Results and discussion

### Performance

We compare the performance of our tools on several fundamental tasks to standard, broadly available software in representative examples and on broadly available computers.

#### Making a mosaic from a huge image

We chose an 8-bit RGB colour JPEG-compressed TIFF file of 103168 ×63232 pixels originating in the digitization of a pathology slide. The original file weighted 975.01 MiB. Loading this image entirely into RAM would need at least 3×103168×63232=18.2 GiB and is presently intractable on most if not all desktop and laptop computers of reasonable cost.

The task was to produce, from this image, a mosaic of 64 pieces so that each one needs less than 512 MiB RAM to open.

On a 3.2 GHz Intel Core i3 IMac computer with 16 GB of RAM, the convert command from ImageMagick (version 6.8.0-7 with quantum size 8 bits) was unable to complete the request. GraphicsMagick (gm convert-crop; version 1.3.17 with quantum size 8 bits) completed the request in 70 min, using 25 GiB of disk space. tiffmakemosaic from our LargeTIFFTools completed the request in 2.5 min.

To ascertain that this task can be equally achieved even on computers with a modest RAM amount, we performed the same task on a 6-year-old 2.66 GHz Core2Duo Intel IMac with 2 GiB RAM. The task was completed in 9.0 min.

#### Converting NDPI into TIFF

*Splitting a NDPI file into TIFF files.* A pathology sample (6.7 cm^2^ of tissue) was scanned at magnification 40x and with 11 focus levels (every 2 microns) by a NanoZoomer, resulting in a 6.5 GiB file in proprietary NDPI format (called file a.ndpi hereafter). On a 2.6 GHz Intel Core i7 Mac Mini computer with 16 GiB RAM, ndpisplit extracted all 55 images (11 focus levels and 5 magnifications) as independent, single-image TIFF files with JPEG compression in 7.11 min. The size of the largest images was 180224×70144. The speed was limited only by the rate of I/O transfers since the CPU usage of this task was 1.38 min, out of which the system used 1.30 min. Executing again the same task straight after the first execution took only 0.57 min because the NDPI file was still in the cache of the operating system.

To ascertain that this task can be equally achieved even on computers with a modest RAM amount, we made a try on a 6-year-old 2.66 GHz Core2Duo Intel PC with 2 GiB RAM running 32-bits Windows XP Pro SP3. The original file shown in Figure 1, called b.ndpi, and weighting 2.07 GiB (largest image: 103168×63232 pixels), was split into independent TIFF files in 2.2 min without swapping.

In comparison, the LOCI Bio-Formats plugins for ImageJ [25], in its version 4.4.6 with ImageJ 1.43 m, was not able to open the images in file a.ndpi even at low resolution.

*Converting a NDPI file into a multiple-images TIFF file.* Alternatively, the same proprietary-format file a.ndpi was converted into a multiple-images TIFF file with ndpi2tiff. On the same computer as before, the conversion time was 7.0 min. Here again, the speed of the process is limited only by the rate of I/O transfers since the conversion took only 30 s if performed when the NDPI file was still in the cache of the operating system.

Since the resulting TIFF file could not store all 55 images in less than 4 GiB, we passed the option -8 on the command line to ndpi2tiff to request using the BigTIFF format extension. The specifications of this extension to the TIFF standard, discussed and published before 2008 [33,34], are supported by LibTIFF as of version 4.0.0 [27], and therefore by the abundant image viewing and manipulation software which relies on LibTIFF. If the use of the BigTIFF format extension would have impeded the further exploitation of the produced TIFF file, we could have simply used ndpisplit as above. Or we could have called the ndpi2tiff command several times, each time requesting extraction of a subset of all images by specifying image numbers after the file name, separated with commas, as in a.ndpi,0,1,2,3,4.

#### Extracting a small region from a huge image

This task can be useful to visualize at full resolution a region of interest which the user has selected on a low-magnification preview image. Therefore, it should be performed as quickly as possible.

#### From a TIFF file

The task was to extract a rectangular region of size 256×256 pixels situated at the bottom right corner of huge TIFF images and to save it as an independent file. The source images were single-image TIFF files using JPEG compression. Table 1 compares the time needed to complete the task with tifffastcrop from our LargeTIFFTools and with several software tools, on increasingly large TIFF files. Tests were performed on a 2.6 GHz Intel Core i7 Mac Mini computer with 16 GB of RAM and used GraphicsMagick 1.3.17, ImageMagick 6.8.0-7 and the utility tiffcrop from LibTIFF 4.0.3. Noticeably, when treating the largest image, GraphicsMagick needs 50 GiB of free disk space, whereas tifffastcrop doesn’t need it.

**Table 1:** **Speed comparison of software to extract a *256×256 * rectangle from a huge TIFF image**

**Image size (px)**	***11264×4384***	***45056×17536***	***180224×70144***
tifffastcrop	0.30 s	0.30 s	0.30 s
GraphicsMagick	0.74 s	23.6 s	>80 min
ImageMagick	1.18 s	236 s	failed
tiffcrop	0.50 s	failed	seg. fault

Time needed (or indication of failure when the task was not completed) by several software tools to extract a rectangular region of size ***256×256*** pixels situated at the bottom right corner of huge TIFF images, and to save it as an independent file. The input images were single-image tiled TIFF files using JPEG compression. Their dimensions are indicated in the top row. The computer used was a 2.6 GHz Intel Core i7 Mac Mini with 16 GiB of RAM and more than 100 GiB of free hard disk. The tested software tools were, from top to bottom, tifffastcrop from our LargeTIFFTools, GraphicsMagick 1.3.17, ImageMagick 6.8.0-7 and the utility tiffcrop from LibTIFF 4.0.3.

#### From a NDPI file

The task was to extract a rectangular region of size 256×256 from one of the largest images of the file a.ndpi (size 180224×70144). On a 2.6 GHz Intel Core i7 Mac Mini computer with 16 GB of RAM, the execution time was 0.12 s for one extract, and in average 0.06 s per extract in a series of 20 extracts with locations drawn uniformly at random inside the whole image.

### Applications

#### Integration in digital pathology image servers or virtual slide systems

The NDPITools are being used in several other software projects: 

•in a system for automatic blur detection [2,4].

•in WIDE [22], to deal with NDPI files. WIDE is an open-source biological and digital pathology image archiving and visualization system, which allows the remote user to see images stored in a remote library in a browser. In particular, thanks to the feature of high-speed extraction of a rectangular region by ndpisplit, WIDE saves costly disk space since it doesn’t need to store TIFF files converted from NDPI files in addition to the latter.

#### Exploiting a large set of digital slides

In the framework of a study about invasive low-grade oligodendrogliomas reported elsewhere [8], we had to deal with 303 NDPI files, occupying 122 GiB. On a 3.2 GHz Intel Core i3 IMac computer with 16 GB RAM, we used ndpisplit in a batch work to convert them into standard TIFF files, which took only a few hours. The experimental -s option of ndpisplit was used to remove the blank filling between scanned regions, resulting in an important disk space saving and in smaller TIFF files (one for each scanned region) which where easier to manipulate afterwards. Then, for each sample, Preview.app and ImageJ were used to inspect the resulting images and manually select the regions of clinical interest. The corresponding extracts of the high magnification images were the subject of automated cell counting and other quantitative analyses using ImageJ. In particular, we collected quantitative data about edema or tissue hyperhydration [8]. This quantity needed a specific image analysis procedure which is not offered by standard morphometry software and, unlike cell density estimates, could not be retrieved by sampling a few fields of view in the microscope. Therefore, virtual microscopy and our tools were essential in this study.

#### Study of a whole slide of brain tissue invaded by an oligodendroglioma

To demonstrate the possibility to do research on huge images even with a modest computer, we chose a 3-year-old MacBook Pro laptop computer with 2.66 GHz Intel Core 2 Duo and 4 GiB of RAM. We used ImageJ and the NDPITools to perform statistics on the upper piece of tissue on the slide shown in Figure 1.

Since the digital slide b.ndpi weighted 2.07 GiB, with a high resolution image of 103168×63232 pixels, it was not possible to do the study in a straightforward way. We opened the file b.ndpi as a preview image with the command Plugins > NDPITools > Preview NDPI... and selected on it the left tissue sample. Then we used the command Plugins > NDPITools > Custom extract to TIFF / Mosaic... and asked for extraction as a mosaic of 16 JPEG files, each one needing less than 1 GiB of RAM to open, and with an overlap of 60 pixels. This was completed within a few minutes. Then we applied an ImageJ macro to each of the 16 pieces to identify the dark cell nuclei (those with high chromatin content), based on thresholding the luminosity values of the pixels, as shown in Figure 1. It produced text files with the coordinates and size of each cell nucleus.

Out of the 154240 identified nuclei, 1951 were positioned on the overlapping regions between pieces. Using the overlap feature of our tools enabled to properly detect these nuclei, since they would have been cut by the boundary of the pieces of the mosaic in absence of overlap. We avoided double counting by identifying the pairs of nuclei situated in the overlapping regions and which were separated by a distance smaller than their radius.

As shown in earlier studies [7,10,11], these data can be used for research and diagnosis purposes. As an example, Figure 5 shows the distribution of the distance of each cell nucleus to its nearest neighbor. Thanks to the very high number of analyzed cell nuclei, this distribution is obtained with an excellent precision.

**Figure 5:** The positions of the 154240 identified nuclei were obtained from the analysis with ImageJ of the digital slide on a laptop computer. Since the slide was too large to fit into the computer’s memory, it was turned into a mosaic of 16 pieces with overlap of 60 pixels, and each piece underwent automated analysis independently. Then the results were aggregated. The graph shows the probability density function of the distance of a cell nucleus to its nearest neighbor in the whole sample.

## Conclusions

The LargeTIFFTools, NDPITools and NDPITools plugins for ImageJ achieve efficiently some fundamental functions on large images and in particular digital slides, for which standard open source software fails or performs badly. They enable both the clinician to examine a single slide and the bioinformatics research team to perform large-scale analysis of many slides, possibly on computer grids [20].

To date, the LargeTIFFTools have been downloaded from more than 388 different IP addresses, the NDPITools from more than 1361 addresses, and the ImageJ plugins from more than 235 addresses. Table 2 lists the distribution of the target platforms among the downloads of the binary files. It shows a broad usage of the different platforms by the community, emphasizing the importance of cross-platform, open source tools.

**Table 2:** Downloads of the NDPITools

**Windows (32 bits)**	**Windows(64 bits)**	**Linux**	**Mac OS X**
483	542	217	285

Distribution of the downloads (unique IP address) of the precompiled binaries of the NDPITools between March 2012 and April 2013.

We have explained how the software was used to study some microscopic properties of brain tissue when invaded by an oligodendroglioma, and we have given an illustrative application to the analysis of a whole-size pathology slide. This suggests other promising applications.

## Availability and requirements

a. LargeTIFFTools 

•**Project name:** LargeTIFFTools

•**Project home page:**http://www.imnc.in2p3.fr/pagesperso/deroulers/software/largetifftools/

•**Operating system(s):** Platform independent

•**Programming language:** C

•**Other requirements:** libjpeg, libtiff

•**License:** GNU GPLv3

b. NDPITools 

•**Project name:** NDPITools

•**Project home page:**http://www.imnc.in2p3.fr/pagesperso/deroulers/software/ndpitools/

•**Operating system(s):** Platform independent

•**Programming language:** C

•**Other requirements:** —

•**License:** GNU GPLv3

For the convenience of users, precompiled binaries are provided for Windows (32 and 64 bits), Mac OS X and Linux.

c. NDPITools plugins for ImageJ 

•**Project name:** NDPITools plugins for ImageJ

•**Project home page:**http://www.imnc.in2p3.fr/pagesperso/deroulers/software/ndpitools/

•**Operating system(s):** Platform independent

•**Programming language:** Java

•**Other requirements:** ImageJ 1.31s or higher, Ant, JAI 1.1.3

•**License:** GNU GPLv3

## Competing interests

The authors declare that they have no competing interests.

## Authors’ contributions

CD wrote the paper. ML conceived and implemented a first version of the integration into ImageJ as a *toolset* of macros. CD implemented the software and wrote the documentation. CG, AG and ML contributed suggestions to the software. CD, DA, AG and ML performed software tests. CD, MB, CG, AG and ML selected and provided histological samples. CD performed the statistical analysis of the sample slide. All authors reviewed the manuscript. All authors read and approved the final manuscript.
